The article "A Robust Image Encrypted Watermarking Technique for Neurodegenerative Disorder Diagnosis and Its Applications" was retracted in 2023. Reasons: signs of a paper mill; compromised peer review; unreliable results or conclusions.

# A Robust Image Encrypted Watermarking Technique for Neurodegenerative Disorder Diagnosis and Its Applications

**DOI:** 10.1155/2021/8081276

**Published:** 2021-09-20

**Authors:** Chirag Sharma, Amandeep Bagga, Rajeev Sobti, Mohammad Shabaz, Rashid Amin

**Affiliations:** ^1^Department of Computer Science and Engineering, Lovely Professional University, Punjab, India; ^2^Department of Computer Application, Lovely Professional University, Punjab, India; ^3^Arba Minch University, Ethiopia; ^4^Department of Computer Science and Engineering, Chandigarh University, India; ^5^Department of Computer Science, University of Engineering and Technology, Taxila, Pakistan

## Abstract

The use of Internet technology has led to the availability of different multimedia data in various formats. The unapproved customers misuse multimedia information by conveying them on various web objections to acquire cash deceptively without the first copyright holder's intervention. Due to the rise in cases of COVID-19, lots of patient information are leaked without their knowledge, so an intelligent technique is required to protect the integrity of patient data by placing an invisible signal known as a watermark on the medical images. In this paper, a new method of watermarking is proposed on both standard and medical images. The paper addresses the use of digital rights management in medical field applications such as embedding the watermark in medical images related to neurodegenerative disorders, lung disorders, and heart issues. The various quality parameters are used to figure out the evaluation of the developed method. In addition, the testing of the watermarking scheme is done by applying various signal processing attacks.

## 1. Introduction

The accessibility of multimedia details across the web has caused unintended individuals in distributing information, including videos, illegally. Problems regarding copyright protection as well as ownership identification are actually prominent; also, the improvement of the secured strategy is necessary to fight these problems—electronic patient information and images distributed illegally. The unlawful distribution of multimedia is shown in Figure 1. Thus, a need for an authorized method is required to recognize these unlawful users, thus ending the distribution of content illegally. Healthcare data is also suffering from integrity issues. The requirement of a secured technique is achieved from encryption, steganography, and watermarking. Since watermarking has a broader scope compared to both, we have used watermarking in this paper combined with encryption. All the multimedia data and medical images are watermarked before they are transmitted.

There is a big challenge to embed a watermark in medical images. Watermarking is a technique to embed unnoticeable signal in any multimedia which is not visible to any intruder. The distribution of medical records of the patient is required to be secured before being shared in various sites. Medical images generate a diagnosis of internal parts of human bodies involving multiple organs and tissues. These involve MRI (Medical Resonance Imaging), ultrasounds, endoscopy, thermography [1], etc. Adding the watermark inside medical images introduces the challenge of quality loss, and slight loss of information can impact the diagnosis. So a secured watermarking technique is proposed in this paper to tackle these issues. Medical images are categorized into a CT scan, MRI, NMI, ultrasound, and X-rays. CT scan images are used to find details inside the human body of incredibly soft tissue. MRI (Magnetic Resonance Imaging) is similar to CT scan images, but the higher quality of the image is produced. MRI provides more detailed information regarding the entire body. Nuclear Medical Imaging (NMI) produces a 3D image of the specific parts of the body. Ultrasound images are used to show the movement of the unborn child in real time. X-rays create radiation-based images to find a defective part of the bone. The different formats of medical image formats are NIfTI (Neuroimaging Informatics Technology Initiative), DICOM (Digital Imaging and Communications in Medicine), Joint Picture Expert Group (JPEG), and PNG (Portable Network Graphics).

Figure 1 represents the illegal distribution of multimedia data across the Internet without information of the original user.  Figure 2 explains the process of embedding secret signal inside multimedia data.  Figure 3 describes the various techniques of watermarking in various forms. Watermarking can be categorized in the form of domain, document, perception, and application. We are going to use the invisible watermarking technique on standard images and medical images. COVID-19 has brought many challenges in forging medical records [3], so a robust method is needed to combat the problems in particular in various fields of diagnosis of neurodegenerative disorders, heart diseases, and lung issues. Neurodegenerative disorders are disorders that impact the lifestyle of humans that cause issues in breathing, movement, and talking and heart-related issues. The diagnosis of these disorders is done using various techniques such as nerve conduction studies and electromyography. These techniques are applied to check how much nerve is damaged using electrodes in the body. There are various types of medical images used in the diagnosis of neurodegenerative disorders such as MRI and CT images.

The comparative analysis of existing transformation techniques has been presented in Table 1(a). It has been observed that frequency domain methods have a clear advantage over spatial domain techniques in terms of real-time applications. In the proposed work, we have used graph-based transform as it has excellent data correlation and decorrelation properties; DCT is less adaptable to all types of images. GBT provides good results in residual signals, predicting a good level of difference between the actual and expected output. GBT has better energy compaction and high construction quality properties than DCT and DWT. GBT is known as edge adaptive transform that has good results in edge detection mechanisms.

Table 1(b) represents the comparative analysis of encryption algorithms used in the field of watermarking. The quality loss is actually the study's primary constraint as the watermark's embedding affects medical-related images' quality. There are a lot of watermarking methods offered. The most common types of frequency domain methods are DCT and DWT, which are further combined with other transforms to achieve good results in the field of watermarking [4, 5]. Graph-based transform is used to tackle image compression issues in DCT. Many scientists are putting on these strategies to make an answer to find appropriate watermarking techniques. While these strategies are excellent, improvements may be made in numerous areas. In COVID-19, many unintended users are finding various ways in manipulating information. The websites of hospitals are getting hacked. The patient's record is getting manipulated without information of the owner. The proposed technique will tackle the issues in protecting the patient's records without information of the owner, thus achieving good use in digital rights management (DRM). The encryption mechanism utilized in the proposed scheme contributes to more security features. It will be practically difficult to recognize a watermark from the watermarked content. The developed method in the paper is based on singular value decomposition and graph-based transform. The mechanism of encrypting the watermark is done before watermarking. Embedding an encrypted watermark proposes scrambling the watermark image in a limited time as other mechanisms like DES and AES take a large amount of time for computation. Hence, a fast mechanism that emphasizes selecting certain features and Lyapunov exponents—the encryption on hyperchaos—is used in this analysis. The watermarking technique is evaluated by enforcing a variety of signal processing attacks. The performance parameters used in this research are PSNR, NC, SSIM, and BER. The substantial development done in the manuscript is given below:

- We developed a watermarking method by embedding an encrypted watermark on standard medical images using hyperchaotic encryption, singular value decomposition, and graph-based transform
- We applied signal processing attacks on the proposed method to check the efficiency of the mechanism
- We evaluated results using different quality metrics

Section 2 reviews all of the associated efforts carried out to this specific region.  Section 3 describes the research methodology used in this paper.  Section 4 analyzes the obtained results.  Section 6 describes the conclusion received from the proposed work.

## 2. Review of Literature

Probably the most prominent watermark embedding method will be the Discrete Wavelet Transform (DWT). Many scientists have applied this method as the transformation as DWT is a dependable technique. However, the least significant bit modification process is not substantial to deal with some signal processing attacks [6–8]. Many researchers [9–11] have used frequency domain methods like DCT and DWT [12]. The forms generally face the issue like reduction in the dimensionality of the matrix, that is, the reason these methods had been fused with one other way called singular value decomposition (SVD). The decomposition technique SVD [13, 14] was extracting a significant amount of functions such as the *S* part in a matrix of SVD as it can take care of picture compression, as well as processing strikes as well as the watermark embedding, which will not be influenced when any of the frequency domain techniques are fused with SVD. A multiwavelet video watermarking technique SVD-DWT was introduced [15, 16]. A semiblind SVD-DWT method was developed to be applied on videos of the compressed domain [17].

DWT-SVD [18] is applied on various images, and various researchers proposed a GWO optimizer to encounter convergence issues in optimization algorithms. A hybrid method with the firefly optimization algorithm was developed to get high values [19]. The method SVD-BWT was developed along with optimization [20]. Various dynamic algorithms like PSO, GWO, firefly, and cuckoo search [16, 21–23] improve the existing algorithms' efficiency by targeting high-fitness function values with their respective mathematical model. GBT [24] uses graphs in the form of signals, and this transform is applied for depth map coding [17, 25, 26]. GBT was combined with SVD for pictures of the respective labor [2, 27]. Wang et al. [28] introduced an image encryption mechanism based on multiple chaos. Cao and Wang [29] applied a hyperchaotic encryption mechanism [30] to the watermark embedding technique to ensure more security, and the proposed method provided better results than the transposition cipher used in [31].

## 3. Proposed Methodology

This section proposes a watermark embedding technique on medical, standard images and specific attacks on the proposed method.

### 3.1. Watermarking Technique

The first step would be to embed an encrypted watermark of multimedia information. The addition of a watermark encounters a tremendous issue of loss of quality. The proposed strategy is a hybrid transformation strategy based on singular value decomposition and edge adaptive graph-based transform. The addition of the watermark is carried out by hyperchaotic encryption. The proposed embedding technique is robust enough to counter all signal processing attacks. The edge adaptive GBT transforms the signal in the form of a graph and has much better outcomes in adapting the image's signal structure. SVD counters the dimensionality reduction problems. The selected healthcare impression is transformed by using GBT. The *S* value from SVD is merged with the *S* value of the watermark. The reason to choose the *S* value out of *U*, *S*, and *V* is to withstand specific signal processing attacks that impact multimedia data. It finds areas where the chances of noise are more. It picks most of the information in fewer coefficients after the image transformation to matrix form is done. The *S* value finds high values of robustness against noise attacks. During decomposition, the noise gets separated from the data but stays in orthogonal matrices *U* and *V*. The *S* component deletes most nonzero coefficients in the image.

#### 3.1.1. Graph-Based Transform and Singular Value Decomposition Technique

The representation of graph-based transform is done in *G* = {*M*, *K*, *s*}, where *M*, *K*, and *s* represent vertices, edges, and signal, respectively.

(1) $$\begin{array}{c} T\left(m,n\right)=\left\{\begin{array}{cc} \sum Tm,n, & \text{if }m=n\\ 0, & \text{otherwise} \end{array}\right\}, \end{array}$$

where weight is represented by *T*(*m*, *n*). The diagonal matrix is represented by *Y*(*m*, *n*):

(2) $$\begin{array}{c} Y\left(m,n\right)=\left\{\begin{array}{cc} \sum Ym,n, & \text{if m}=n\\ 0, & \text{otherwise} \end{array}\right\}. \end{array}$$

Then, the Laplacian-graph matrix *L* would be defined as

(3) $$\begin{array}{c} L=T-Y, \end{array}$$

where *L* is the Kirchhoff operator represented by an adjacency matrix. Eigenvalue decomposition is done of real nonnegative eigenvalues **Λ** = {**λ**1, **λ**2, ⋯**λN**}; **V** = {*v*1, ⋯, *vN*} represents orthogonal eigenvectors derived as

(4) $$\begin{array}{c} L=V\Lambda V^{T}, \end{array}$$

(5) $$\begin{array}{c} M=V^{T}s, \end{array}$$

(6) $$\begin{array}{c} \text{SVD}=\overset{r}{\underset{A=1}{\sum }}UB*SB*{\left(VB\right)}^{T}=\overset{r}{\underset{i=1}{\sum }}UM*SM*{\left(VM\right)}^{T}, \end{array}$$

(7) $$\begin{array}{c} UB=\left[u1,u2,u3,u4\cdots uN\right], \end{array}$$

(8) $$\begin{array}{c} VB=\left[v1,v2,v3,v4\cdots vN\right], \end{array}$$

(9) $$\begin{array}{c} S_{y}=\left(\begin{array}{ccc} S_{1} & \cdots & N\\ \vdots & \ddots & \vdots \\ 0 & \cdots & S_{N} \end{array}\right), \end{array}$$

(10) $$\begin{array}{c} \text{SVD}={USV}^{T}, \end{array}$$

(11) $$\begin{array}{c} W^{\prime }\left(m,n\right)=M\left(m,n\right)+\alpha w\left(m,n\right)\;\;. \end{array}$$

#### 3.1.2. Encryption Mechanism on Hyperchaos

A hyperchaotic mechanism is used to encrypt the watermark image *w*(*m*, *n*) before embedding it to a medical image and multimedia data. The advantage of using hyperchaotic encryption lies in its dependency on initial conditions as shown in Figure 4. It provides pseudo-random generation of values after encryption that gives an edge over other algorithms. It involves Lyapunov exponents [2] that ensure that the scrambling does not affect the actual data. The encryption before watermarking is the crucial step as encryption can affect the output data. This encryption ensures that output data is not affected by scrambling and ensures good security levels as it will require a perfect key to decrypt the data. The importance of *w*, *x*, *y*, *z* is estimated from the earlier calculated Lorenz system. The values of *s*, *t*, *u* in scrambling are used [2]. The next step is to find the procedure for scrambling the watermark given in equations (13) and (14). The final action is interchanging the coefficients of *x*(*m*)^th^ row and *m*^th^ row of the picture provided in situations (15), (16), and (17).

(12) $$\begin{array}{c} \left\{\begin{array}{c} x=s\left(y-x\right)+w\\ y=ux-y-xz\\ z=xy-tz\\ w=-yz+rw \end{array}\right\}, \end{array}$$

(13) $$\begin{array}{c} X=\mathrm{mod}\left(\text{floor}\left(x+100\right)*105,m\right)+1, \end{array}$$

(14) $$\begin{array}{c} Y=\mathrm{mod}\left(\text{floor}\left(y+100\right)*105,n\right)+1, \end{array}$$

(15) $$\begin{array}{c} T\left(x,:\right)=T\left(x\left(m\right),:\right), \end{array}$$

(16) $$\begin{array}{c} T1=T, \end{array}$$

(17) $$\begin{array}{c} W1\left(:,n\right)=W1\left(:,y\left(n\right)\right). \end{array}$$

#### 3.1.3. Watermark Extraction

This recovery of the watermark is done using an extraction algorithm. The process of extraction is described in equation (18) and represented in Figure 5.

(18) $$\begin{array}{c} W\left(i,j\right)=\frac{\left(WF^{\prime \left(i,j\;\right)}-A\left(i,j\right)\right)}{\alpha }, \end{array}$$

*w*(*m*, *n*) is the extracted watermark, *W*′(*m*, *n*) is the watermarked image, and *M*(*m*, *n*) is the selected image.

#### 3.1.4. Evaluation of Performance

The technique's performance is measured by evaluation metrics: BER, NC, SSIM, and PSNR. These parameters related the watermarked image to the actual image. The effectiveness of the developed algorithm entirely depends on obtained values of quality metrics. All quality metrics differentiate the original image from the watermarked image to measure the difference between them.

(a) Peak signal to noise ratio (PSNR): PSNR is a tremendous metric to measure that separates watermarked and original pictures based on values of mean square error. This is the particular quality parameter used in the analysis, as it is estimated by complete error. The following situation calculates it:
  (19) $$\begin{array}{c} \text{MSE}=\overset{M-1\;N-1}{\underset{i=0\;j=0}{\sum }}\frac{1}{M*N}{\left(\left[A\left(m,n\right)-E\left(m,n\right)\right]\right)}^{2}, \end{array}$$
  where *M* and *N* represent rows and columns of the image, respectively.
  (20) $$\begin{array}{c} \text{PSNR}=\frac{10\log_{10}{\left(255\right)}^{2}}{\text{MSE}}. \end{array}$$
*A*(*m*, *n*) is the selected image, and *E*(*m*, *n*) is the watermarked image:
  (21) $$\begin{array}{c} \text{Average PSNR}=\frac{\sum_{i}^{n}{\text{PSNR}}_{i}\;}{n}. \end{array}$$
(b) Normalized correlation (NC): this parameter is used to find the correlation between the watermarked image and the selected image. It is calculated by
  (22) $$\begin{array}{c} \text{NC}=\frac{\sum_{i=1}^{G}\sum_{j=1}^{H}\left(A\left(m,n\right)-\bar{A}\right)\left(E\left(m,n\right)-\bar{E}\right)}{\sqrt{\sum_{i}^{G}\sum_{j=1}^{H}{\left(A\left(m,n\right)-\bar{A}\right)}^{2}\sum_{i=1}^{G}\sum_{j=1}^{H}{\left(E\left(m,n\right)-\bar{E}\right)}^{2}}}, \end{array}$$
  where *A*(*m*, *n*) is the selected image, *E*(*m*, *n*) is the watermarked Image, $\bar{A}$ is the mean of selected images, and $\bar{E}$ is the mean of watermarked images.
(c) Structural similarity index measure: this parameter corepresents structural information amongst watermarked and cover images. It is calculated from
  (23) $$\begin{array}{c} \text{SSIM}\left(m,n\right)={\left[l\left(m,n\right)\right]}^{\alpha }{\left[c\left(m,n\right)\right]}^{\beta }{\left[s\left(m,n\right)\right]}^{\gamma }, \end{array}$$
  (24) $$\begin{array}{c} l\left(m,n\right)=\frac{2\mu m\mu n+C1}{\mu^{2}m+\mu^{2}n}, \end{array}$$
  (25) $$\begin{array}{c} c\left(m,n\right)=\frac{2\sigma m\sigma n+C2}{\sigma^{2}m+\sigma^{2}n+C2}, \end{array}$$
  (26) $$\begin{array}{c} s\left(m,n\right)=\frac{\sigma mn+C3}{\sigma m\sigma n+C3}, \end{array}$$
  where *μ*_*m*_, *μ*_*n*_,*σ*_*m*_, *σ*_*n*_, and *σ*_*mn*_ are local means, standard deviation, cross variances of selected frames, and watermarked frames. If *α* = *β* = *γ* = 1 and *C*_3_ = *C*_2_/2, the index simplifies to
  (27) $$\begin{array}{c} \text{SSIM}\left(m,n\right)=\frac{\left(2\mu m\mu n+C1\right)\left(2\sigma m\sigma n+C2\right)}{\left(\mu^{2}m+\mu^{2}n+C1\right)\left(\sigma^{2}m+\sigma^{2}n+C1\right)}. \end{array}$$
(d) Bit error rate: this parameter calculates how much error has occurred after embedding of the watermark. It is inversely proportional to PSNR and is given in the following equation:
  (28) $$\begin{array}{c} \text{BER}=\frac{1}{\text{PSNR}}. \end{array}$$

## 4. Experimental Results

There are approximately 100 MRI medical images, and some standard images have been taken and tested. The images have been obtained from the standard datasets provided by the , Signal and Processing Institute, University of Southern California. The dataset is available for all researchers. Along with these images, encrypted versions of 2 binary watermarks along with watermarks are represented in Figure 6: a total of three standard images and two medical images have been used in this paper. Regular images' names are Bandon, peppers, and fishing boat, and medical images are represented by names medical_1 and medical_2. To achieve the last phase of research, specific quality metrics have been taken. The medical images have been obtained from the open-access medical image repository.

Watermarking is applied to both medical images and normal images. Color image watermarking and greyscale watermarking techniques are used. Color image watermarking is applied to the first three images, and greyscale watermarking is applied to the last two photos.  Table 2 calculates the performance of the proposed technique against no attack. Plots in Figure 7 represent the performance of the embedding technique.

### 4.1. Calculation of Embedding Time

The processing time (in seconds) is estimated in phases of time taken for embedding the specified set of information. The processing time used by the processor is directly proportional to the time taken for embedding. The value of the embedding factor is kept as 0.02. The proposed strategy is quick and, as per processor needs, functions substantially at a very good speed.  Table 3 represents the embedding time of watermarking for various sets of pictures. Plots in Figure 8 presents the complete embedding time taken to embed the watermark.

### 4.2. Processing Attacks

The proposed technique's robustness is tested against a variety of assault scenarios, including Gaussian noise and JPEG compression. The performance of the proposed technique is validated after applying different variance values of attacks. The robustness of the method entirely depends on bit error rate (BER), normalized correlation (NC), structural similarity index measure (SSIM), and peak signal to noise ratio (PSNR). The processing attacks are applied to evaluate the efficiency of the proposed algorithm. The higher value of Gaussian noise and a higher percentage in compression value will impact the quality of the output watermarked image.

#### 4.2.1. Gaussian Noise Attack

Gaussian noise is a white noise attack applied to the selected picture, and also the calculation of outcomes is made appropriately. It can be noticed from plots in Figure 9 that the typical PSNR, NC, and SSIM decrease with growth in encounter worth, and BER improves with an increase in attack.

Table 4 represents calculated values of performance parameters after Gaussian noise attack is applied.

#### 4.2.2. JPEG Compression Attack

A compression value of 96 is put up on selected images and a watermarked and selected image's performance. The lower value of Joint Picture Expert Group (JPEG) compression will impact the quality of the output image.  Table 5 describes calculated performance metric values.  Figure 10 represents plots of watermarking techniques against JPEG compression attack. The compression attack directly impacts the quality of the output watermarked image. The loss compression attack lowers the value of the peak signal to noise ratio when the original image is compared with a compressed watermarked image. We have used a lossless compression attack to calculate results.

## 5. Comparison with Existing Methods

The proposed technique's performance is tested based on two properties: the degree of invisibility and embedding time. Many researchers have researched over the years to improvise on existing mechanisms. This section explains the comparison of the proposed technique against the previous research over the years.  Table 6 compares the proposed method against various techniques based on values of embedding time and quality metrics. Every researcher has used a different dataset of medical images depending upon the requirement; judging the performance of the technique based on quality metrics cannot give the exact version of the performance of the proposed method against existing techniques. The embedding time becomes the crucial factor in comparing the proposed method against existing procedures. The comparison analysis is performed on different sets of images, and the estimation of embedding time is calculated in seconds. It has been concluded that the performance of the watermarking techniques varies for a different collection of images. The embedding time provides the effectiveness of the proposed method. It has been observed from the results presented in Table 6 that our proposed technique performs better than some existing methods in terms of embedding time. The addition of optimization algorithms [22, 32–43] to the proposed approach can positively impact high values of quality metrics (PSNR).

It has been observed from plot in Figure 11 that our proposed technique achieves good results in embedding time. However, the quality issues can persist as the values of PSNR can still be improved by the addition of an optimization algorithm [32–43]. Higher values of PSNR indicate good levels of robustness.

## 6. Conclusion and Future Work

A novel medical-related image watermarking method was developed to enhance security in the field of medical applications. The hybrid mixture of graph-based transform, singular value decomposition, and hyperchaotic encryption gives effective embedding of watermark advantages. The proposed technique was applied in standard and medical images. The additional security mechanism, hyperchaotic encryption, is used in the proposed work and covers the security of both types of images. The proposed technique finds its application in the field of healthcare. The image's quality is not altered after the addition of the watermark, and results indicate the proposed technique's good performance. The proposed method is fast, and the addition of an optimization algorithm will improve the value of quality metrics. Higher values of quality metrics can still be targeted by adding various metaheuristic algorithms such as Ant Colony Optimization (ACO), Grey Wolf Optimization (GWO), and firefly algorithm. The addition of optimization algorithms will improve the values of the quality parameter PSNR that will be listed in future work.

## Figures and Tables

**Figure 1:** Unlawful transmission of videos [2].

**Figure 2:** Watermarking method [2].

**Figure 3:** Watermarking techniques [2].

**Figure 4:** Embedding of the watermark.

**Figure 5:** Extraction of watermark.

**Figure 6:** (a–i) (a) Bandon, (b) peppers, (c) fishing boat, (d) medical_1 and (e) medical_2, (f) original watermark1, (g) original watermark2, (h) scrambled watermark1, and (i) scrambled watermark2.

**Figure 7:** (a–d) Plot of quality metrics for images taken in the proposed work.

**Figure 8:** Embedding time of given images.

**Figure 9:** (a–d) Plot of quality metrics for images taken in the proposed work against Gaussian noise attack.

**Figure 10:** (a–d) Plot of quality metrics for images taken in the proposed work against Gaussian noise attack.

**Figure 11:** Plot of comparison analysis of proposed and existing techniques in terms of PSNR and embedding time.

**Algorithm 1:** Watermark addition algorithm.

**Algorithm 2:** Extraction of the watermark.

**Table:** (a) Comparative analysis of existing transform techniques

Domain transform techniques	Robustness	Complexity	Transient signal changes	Edge adaptive transform	Real-time application
LSB	✗	✗	✗	✗	✗
DWT	✓	✓	✓	✗	✓
DCT	✓	✓	✓	✗	✓
DFT	✓	✓	✓	✗	✓
SVD	✓	✓	✓	✗	✓
GBT	✓	✓	✓	✓	✓

**Table:** (b) Various encryption and security techniques used in watermarking

SNO	Name	Functionality
1.	Transposition cipher	This type of cipher comes in the category of simple encryption, where the shifting of plain texts is done in some regular pattern to form the ciphertext
2.	Rail-fence cipher	It is a form of transposition cipher where plain text is scrambled more straightforwardly, and alphabets are written in a zig-zag manner where individual rows are combined to form the ciphertext
3.	AES	It is termed as advanced encryption standard. It is a cipher used to protect classified data and is used on both hardware and software to encrypt sensitive data
4.	DES	It is known as data encryption standard. It is a cipher that is used to encrypt data in blocks of size 64 bits each
5.	RSA	It is known as Rivest–Shamir–Adleman. It is used for specific security services that enable public-key encryption to secure sensitive data
6.	Triple DES	3DES is an enhancement of DES; it has 64-bit block size with 192-bit key size. It is the same as DES but is applied three times more to get more encryption
7.	Hyperchaotic encryption	The hyper chaotic encryption is a modified encryption standard applied to images. It works on predefined values

**Table 2:** Values of quality metrics for selected images.

Image	PSNR	SSIM	NC	BER
Bandon	37.50	0.978	0.993	0.0266
Peppers	37.65	0.976	0.994	0.0265
Fishing boat	38.64	0.966	0.995	0.0258
Medical_1	37.27	0.978	0.999	0.0268
Medical_2	35.32	0.978	0.999	0.0283

**Table 3:** Embedding time for embedding the watermark.

Image	Embedding time (in seconds)
Bandon	1.2314
Peppers	1.3288
Fishing boat	1.2753
Medical_1	1.2456
Medical_2	1.2766

**Table 4:** Values of quality metrics after Gaussian attack.

Image	PSNR	SSIM	NC	BER
Bandon	34.50	0.967	0.992	0.0289
Peppers	36.65	0.965	0.993	0.0272
Fishing boat	37.54	0.956	0.994	0.0266
Medical_1	35.57	0.958	0.998	0.0281
Medical_2	34.22	0.970	0.998	0.0292

**Table 5:** Values of quality metrics after compression attack.

Image	PSNR	SSIM	NC	BER
Bandon	35.40	0.969	0.992	0.0282
Peppers	35.65	0.967	0.994	0.0280
Fishing boat	35.74	0.952	0.992	0.0279
Medical_1	35.87	0.959	0.998	0.0278
Medical_2	35.22	0.973	0.998	0.0283

**Table 6:** Comparison analysis of the proposed method with existing methods in terms of embedding time and PSNR.

Techniques used	PSNR (dB)	Embedding time (in seconds)
Khare and Srivastava [44]	59.43	4.337
Agarwal et al. [16]	36.30	8.062
Sharma et al. [45]	52.57	251.79
Proposed technique	38.64	1.275

## Data Availability

The data shall be made available on request.
